RETRACTED

# Comparison of the Effects of Repeated Applications of Platelet-Rich Plasma versus Platelet-Poor Plasma on Fat Graft Survival in Nude Mice

**DOI:** 10.1155/2021/6613783

**Published:** 2021-02-16

**Authors:** Junjie Li, Wei Chen, Xiao Shi, Pijun Yu

**Affiliations:** ^1^Department of Aesthetic Plastic Surgery, Shanghai Eighth People's Hospital, Shanghai 200235, China; ^2^Department of Anesthesia, Renji Hospital, School of Medicine, Shanghai Jiao Tong University, Shanghai 200240, China

## Abstract

Autologous fat grafting has been widely used for soft tissue filling in plastic surgery. Platelet-rich plasma (PRP) could play a wide role in health and disease because of containing a variety of growth factors and cytokines. Although previous studies have described the positive effect of autologous PRP mixed with fat grafts, only minimal improvements in fat graft survival have been reported. The present study is aimed at comparing the effects of PRP and platelet-poor plasma (PPP) on the survival and quality of fat grafting. We built a 180-day nude mouse model implanted with a fat graft supplemented with PRP, PPP, or saline, respectively. The above reagents (PRP, PPP, or saline) were injected two additional times after the initial engraftment. The survival ratio of the fat grafts and the capillary density in the PRP group were significantly higher than those in the PPP group and the saline group (control group) at 15, 30, 90, and 180 days posttransplantation (*P* < 0.05). The survival ratio of the PPP group was higher than that of the saline group (*P* < 0.05), but the capillary density in the PPP group was not significantly different from that in the saline group at any time point (*P* > 0.05). We hence conclude that the repeated application of PRP or PPP three times can enhance the survival of fat grafts within 180 days. Moreover, the effect of PRP is superior to that of PPP.

## 1. Introduction

Autologous fat grafting has been extensively used to fill soft tissue in plastic and reconstructive surgery since it was first described by Neuber in 1893 [1–3]. Autologous fat grafting has many potential advantages over other methods of soft tissue augmentation: nonimmunogenic, biocompatible, abundant, easily harvested, and of natural physiological characteristics [4–6]. However, the low and unpredictable survival rate of grafts remains a primary challenge, as reported in many experimental and clinical studies [7, 8]. In addition, fat grafting is also associated with numerous negative complications, including liquefaction, necrosis, calcification, and the formation of cysts [9].

Platelet-rich plasma (PRP) is defined as the portion of the plasma fraction of whole blood that has a high platelet concentration above the baseline level [10, 11]. When activated by factors such as thrombin or calcium, alpha granules of the platelets could release various growth factors and cytokines such as platelet-derived growth factor (PDGF), transforming growth factor-*β* (TGF-*β*), vascular endothelial growth factor (VEGF), insulin-like growth factor (IGF), fibroblast growth factor-2 (FGF-2), and epidermal growth factor (EGF) [12, 13]. The use of PRP has been described for a wide variety of clinical applications, particularly in craniomaxillofacial surgery, spine and joint arthroplasty, periodontal surgery, and wound healing [14–18]. Previous studies have demonstrated positive effects of PRP, supporting its clinical use. In contrast, platelet-poor plasma (PPP) has a lower concentration of platelets than PRP [19, 20]. Zhang et al. [21] confirmed that PPP maintained the phenotype of osteoblastic cells and enhanced the rate of MSC proliferation. However, few studies have attempted to evaluate the effects of PPP on fat grafting.

RETRACTED

To overcome the drawbacks of fat grafting alone, several studies have described the major effects of the combination of autologous PRP and fat grafts [15, 22]. For example, Hersant et al. [23] evaluated the effects of PRP on resorption and adipocyte survival in autologous fat grafts in rats. Although the documented results indicated that the application of PRP enhanced the survival and quality of fat grafts, the degree of improvement reported in previous studies was not significant because fat grafting was combined with only one application of PRP, and PRP was quickly absorbed during the early posttransplantation phase.

In this study, to better improve the survival and quality of fat grafting, we combined *in vivo* fat grafts with PRP, PPP, or saline, respectively. The treatment solution was administered three times, and the effects of PRP and PPP on the transplant were compared.

## 2. Materials and Methods

### 2.1. Experimental Animals

Thirty-six 5-week-old female BALB/c nude mice weighing 19-22 g were obtained from the Shanghai SLAC Laboratory Animal Co., Ltd. (Shanghai, China). The mice were maintained on a standard laboratory diet with water provided ad libitum. The use of animals in this study and our experimental protocols were approved by the Institutional Animal Care and Use Committee at Shanghai Eighth People's Hospital (Shanghai, China).

### 2.2. Isolation and Preparation of Human Fat Tissue

Under local anesthesia, fat tissue was harvested from the lateral thigh of a 25-year-old healthy woman using a 2 mm diameter blunt cannula attached to a 10 mL Luer-Lok syringe (Becton Dickinson Co., NJ, USA) under manual regulation of negative pressure. The aspirated fat was washed with 0.9% sodium chloride solution (saline), held in the syringe vertically for 3 minutes, and then separated into three layers (the upper layer was composed of oil, the middle layer was composed of adipose tissue, and the lower layer was composed of blood). The upper and lower layers were discarded. The procedure above was repeated three times to obtain 60 mL of purified fat. The participant provided informed consent, and an institutional review board-approved protocol was used.

RETRACTED

### 2.3. Preparation of PRP and PPP

Blood (40 mL) was drawn from the same donor's cubital vein using a 50 mL syringe that contained 10% sodium citrate as an anticoagulant and then equally divided into four 15 mL sterile tubes (Corning, Inc., NY, USA). The blood aliquots were centrifuged twice at 200 × *g* for 10 minutes at 20°C. The blood was first centrifuged at 200 × *g* for 10 minutes using an Eppendorf 5810R centrifuge (Eppendorf AG, Hamburg, Germany), and the supernatant, including the buffy coat and 1 mm below the buffy coat, was decanted into four other sterile 15 mL tubes. The second centrifugation step was performed at 200 × *g* for 10 minutes. The top 1 mL portion of the supernatant was taken as the PPP, and the bottom 1 mL portion was collected as the PRP. The platelet concentrations in the PRP, PPP, and whole blood were determined using a Sysmex KX-21N (TOA Medical Electronics Co., Kobe, Japan) hematology analyzer (PRP: 1058.33 × 10^9^ ± 37.740 platelets/L, PPP: 34.12 × 10^9^ ± 6.014 platelets/L, and whole blood: 223.00 × 10^9^ ± 11.136 platelets/L). Finally, 0.1 mL of 10% calcium chloride (Sigma-Aldrich Co., California, USA) was added to aliquots of 1 mL PRP and 1 mL PPP and stored at 4°C for 12 hours to induce platelet activation and exocytosis of the alpha granules.

### 2.4. Animal Model and Groups

Thirty-six nude mice were randomly divided into the PRP group, the PPP group, and the saline group (control group) with 12 mice per group. The subcutaneous dorsal layers of the right and left sides of each mouse were designated as the two recipient regions for fat graft transplantation. While the mouse was manually restrained, 0.8 mL of a combination of fat and PRP (10 : 2), fat and PPP (10 : 2), or fat and saline (10 : 2) was injected into the PRP, PPP, or saline recipient region, respectively, with a 2 mm diameter blunt cannula (Figure 1(a)). At 5 and 10 days after the first transplantation, 0.14 mL of PRP, PPP, or saline was injected into each respective fat graft of the three groups with 1 mL syringes. At 15, 30, 90, and 180 days after the first transplantation, three mice from each group were randomly selected and sacrificed. Transplant specimens were harvested and analyzed as described below (Figure 1(b)).

RETRACTED

### 2.5. Macroscopic Examination

All transplants from each group were dissected, and the survival weight and volume were measured. The weight was determined using an electronic balance (Ohaus Co., NJ, USA), and the volume was measured by the amount of water displaced inside a test tube [24]. A transverse section of each transplant was examined macroscopically for two parameters: liquefaction and necrosis. The parameters were graded on a semiquantitative scale of 0-2 for each transplant as follows: 0 = absence of liquefaction and necrosis, 1 = liquefaction, and 2 = necrosis.

### 2.6. Histological Examination

The transplants were fixed in a 10% formaldehyde solution for 24 hours, embedded in paraffin, and then sectioned in 5 *μ*m increments along the axis perpendicular to the longest axis of the transplant. One section of the maximum area per graft was stained with hematoxylin-eosin (HE) and examined under a light microscope (Olympus Co., Japan) in each group. For each section, the histological parameters that were identified included viable adipocytes, cysts, vacuoles, necrosis, and blood vessels. The necrosis area ratio (including the cyst and vacuole area) was determined by point counting [25] using digital video imaging (JVC TK-C1480E) in adjacent and nonoverlapping fields along any one axis of each HE-stained slide (magnification, ×40). Neovascularization was assessed by counting the capillaries in three adjacent and nonoverlapping fields beginning from the tissue membrane along any one axis of each HE-stained slide (magnification, ×100). Counting was performed by two blinded reviewers.

### 2.7. Assessment of Available Fat Graft Survival

The available survival ratio of each fat graft was determined by combining the aspect of macroscopical volume with the aspect of microhistology, which was calculated using the following equation (survival volume: the volume of each dissected transplant, previous volume: the volume of the fat part of each combination):

(1) $$\begin{array}{c} \text{Previous volume }\left(\text{mL}\right)=0.8\times \frac{10}{10+2},\\ \text{Available survival ratio of the fat graft }\left(\%\right)=\frac{\text{Survival volume}}{\text{Previous volume}}\times \left(1-\text{Necrosis area ratio}\right)\times 100\%. \end{array}$$

### 2.8. Statistical Analysis

Results are expressed as the mean ± standard deviation. The treatment groups were compared using one-way analysis of variance (ANOVA), and multiple comparisons were performed using the least significant difference (LSD) test. *P* values < 0.05 were considered statistically significant. The Kruskal-Wallis *H* test was only used to compare the liquefaction and necrosis grades of the transverse sections, and the statistical significance was set at *P* < 0.016. All data were analyzed using SPSS for Windows version 19.0.

RETRACTED

## 3. Results

### 3.1. Macroscopic Analysis

All nude mice tolerated the procedure without death or complications and were healthy at the time of tissue harvesting. There was no gross indication of acute infection, inflammation, abscess formation, or seroma on the graft itself or on the adjacent host tissues in any mouse. The liquefaction and necrosis grades of the transverse sections in the PRP group were much better than those in the saline group at all time points (*P* < 0.016), but no statistically significant differences were found between the PRP group and the PPP group or between the PPP group and the saline group (*P* > 0.016; Figure 2).

### 3.2. Survival Weight and Volume of the Fat Grafts

The survival weight and volume of fat grafts in the PRP group were significantly greater than those in the PPP group and the saline group at 15, 30, and 90 days (*P* < 0.05), but there were no statistically significant differences between the PPP group and the saline group (*P* > 0.05). The fat graft weight and volume of the PRP group and the saline group were significantly greater than those of the PPP group at 180 days (*P* < 0.05); however, no statistically significant differences were observed between the PRP group and the saline group at 180 days (*P* > 0.05; Figure 3).

### 3.3. Necrosis Area Ratio

A significantly lower necrosis area ratio was observed in the PRP group than in the saline group at 15 days (*P* < 0.05), but there were no statistically significant differences in the necrosis area ratio between the PRP group and the PPP group at 15 days (*P* > 0.05). The PRP group had a much lower necrosis area ratio than the PPP group and the saline group at 30, 90, and 180 days (*P* < 0.05), and the PPP group demonstrated a lower necrosis area ratio than the saline group at all time points (*P* < 0.05; Figures 4 and 5).

### 3.4. Capillary Density

The capillary density in the PRP group was much higher than that in the PPP group and the saline group at all time points (*P* < 0.05). However, the capillary density in the PPP group did not significantly differ from that in the saline group at any time point (*P* > 0.05; Figures 5 and 6).

### 3.5. Available Survival Ratio of the Fat Grafts

The available survival ratio in the PRP group was much higher than that in the PPP group and the saline group at all time points (*P* < 0.05). In addition, the survival ratio in the PPP group was higher than that in the saline group at each time point (*P* < 0.05; Figure 7).

RETRACTED

## 4. Discussion

The current study describes a protocol of multiple applications of PRP and PPP (three times) into a fat graft in a nude mouse model. The major findings show that the available survival ratio and capillary density of the fat grafts in the PRP group were much higher than those in the PPP group.

Pires Fraga et al. [26, 27] studied the effect of PRP on the survival of free fat grafts in a rabbit model and demonstrated that the application of autologous PRP could enhance free fat graft survival. Blumenschein et al. [28] also confirmed the efficacy of fat grafts prepared with PRP in maintaining graft volume and survival in a rat model. Cervelli et al. [29, 30] used 0.3-0.5 mL PRP mixed with 1 mL centrifuged fat tissue for reconstructing the face contour and restoring the superficial density of facial tissues, and the examinations after 18 months showed excellent aesthetic improvement. Unfortunately, Lynch and Bashir [31] concluded that PRP did not enhance free fat graft survival in nude mice. However, in all previous studies, PRP was combined with a fat graft only at the time of implantation; thus, PRP was absorbed quickly during the early posttransplantation phase, reducing the effect of PRP on the graft.

In this study, we describe a protocol of repeated application of PRP or PPP into the fat graft three times, with the first application at implantation to produce a relatively high and steady concentration of PRP and PPP for supporting adipocytes. Furthermore, the effects of these treatments on the available survival ratio of the fat graft, the gross weight, the gross volume, and the histologic necrosis percentage were evaluated. Although the survival weight and volume results showed that there were no significant differences between the PRP group and the saline group at 180 days, we found that the PRP group had a much lower necrosis area ratio than the saline group under histological observations at 180 days. Therefore, the available survival ratio, which combines gross and histological aspects, objectively and accurately revealed the maintenance of the fat grafts.

Early and adequate neovascularization is very important for maintaining the viability of a fat graft [32]. Inhibition of the revascularization of a graft reduces graft volume retention and impairs cellular functions [33]. Many growth factors and cytokines including VEGF [34], PDGF [35], FGF-2 [36], EGF [37, 38], and erythropoietin (EPO) [39, 40] have been shown to enhance the vascularization of fat transplantation. PRP contains a variety of natural growth factors [13, 41, 42]. Bir et al. [43] concluded that the sustained release of PRP restored blood perfusion presumably by stimulating angiogenesis, arteriogenesis, and vasculogenesis, in a mouse hindlimb ischemia model. Xiong et al. [44] evaluated the effect of activated PRP on human graft quality and survival in nude mice and demonstrated that PRP enhanced the vascularization of the graft. In contrast, a study by Rodriguez-Flores et al. [45] showed that an isolated fat graft and a fat graft with PRP did not exhibit significant differences in revascularization or the presence of vessels between infiltrated fat cells in a rabbit model. In our study, capillary density in the PRP group was much higher than that in the PPP group at all time points. By comparing the PRP and PPP groups, we demonstrated that PRP could enhance the vascularization of a fat graft during the early posttransplantation phase.

RETRACTED

Except for growth factors, both PRP and PPP contain essential nutrients for cell survival. The addition of PRP or PPP to fat grafts plays an important role in temporary nutrition. In doing so, PRP enhances the viability of adipocytes and enhances the opportunity for angiogenesis. This is particularly important for adipocytes located in the central region of fat grafts, where the environment is ischemic at the initial transplantation. However, this mechanism of nutritional action has not been described in previous works of literature. In our study, both the necrosis area ratio and the available survival ratio in the PPP group were higher than those in the saline group at all time points. In contrast, the capillary density data illustrated that there were no significant differences between the two groups at any time point. Therefore, we suggested that both PPP and PRP may enhance the survival of fat grafts via a mechanism that involves providing the nutritional function of the essential nutrients by repeated application especially in the early stage. Over time, neovascularization has become a leading function to maintain the grafts in the PRP group rather than the PPP group.

Fat grafts contain a certain number of adipose-derived stem cells (ADSCs). Another potential mechanism by which PRP improves fat grafting is to promote the proliferation of ADSCs and the differentiation of ADSCs into adipocytes [44, 46]. Naderi et al. [47] demonstrated that PRP improved the maintenance and function of adipose tissue grafts, which was achieved by stimulating ADSC proliferation. Finally, inflammatory mechanisms cannot be ignored. Rodriguez-Flores et al. [45] reported that the implantation of fat tissue plus PRP induced a lower inflammation than the implantation of fat tissue alone. However, due to the restriction in obtaining abundant fat and blood samples from the same donor, a major limitation of our study is that the sample size was small. Moreover, the available statistics from a period of 180 days indicate that the survival ratio of the fat grafts in the three groups exhibited a downward trend. Therefore, a longer observation period and adjustments to the ratio of PRP to fat graft tissue and the frequency of PRP supplementation are needed.

RETRACTED

## 5. Conclusions

The present study confirms that the repeated application of PRP or PPP to a fat graft three times can enhance the survival of fat grafts within 180 days. Furthermore, the effect of PRP is better than that of PPP.

## Figures and Tables

**Figure 1:** (a) After the first injection of the combination of fat and PRP in the PRP group. (b) Appearance of the fat grafts in the PRP group at 15 days.

**Figure 2:** General observations of fat grafts from the PRP, PPP, and saline groups after the grafts were harvested from mice at 15 days (a), 30 days (b), 90 days (c), and 180 days (d). General observation of the cross-section of fat grafts at 180 days (e).

**Figure 3:** (a) Comparison of the survival weights of the fat grafts in the PRP, PPP, and saline groups (^∗^*P* < 0.05, ^∗∗^*P* < 0.01, and ^#^*P* > 0.05; *n* = 6). (b) Comparison of the survival volumes of the fat grafts in the PRP, PPP, and saline groups (^∗^*P* < 0.05, ^∗∗^*P* < 0.01, and ^#^*P* > 0.05; *n* = 6).

**Figure 4:** Comparison of the necrosis area ratios in the PRP, PPP, and saline groups (^∗^*P* < 0.05, ^∗∗^*P* < 0.01, and ^#^*P* > 0.05; *n* = 6).

**Figure 5:** Histological observations of fat transplants from the PRP (a, d, g, j), PPP (b, e, h, k), and saline (c, f, i, l) groups at 15 days (a–c), 30 days (d–f), 90 days (g–i), and 180 days (j–l) stained with hematoxylin-eosin and imaged with a light microscope (magnification, ×100).

**Figure 6:** Comparison of the capillary densities in the PRP, PPP, and saline groups (^∗^*P* < 0.05, ^∗∗^*P* < 0.01, and ^#^*P* > 0.05; *n* = 6).

**Figure 7:** Comparison of the available survival ratios of the fat grafts in the PRP, PPP, and saline groups (^∗^*P* < 0.05, ^∗∗^*P* < 0.01, and ^#^*P* > 0.05; *n* = 6).

## Data Availability

Some or all data, models, or code generated or used during the study are available from the corresponding author by request.
